# Electroacupuncture Improves Intestinal Dysfunction in Septic Patients: A Randomised Controlled Trial

**DOI:** 10.1155/2018/8293594

**Published:** 2018-06-26

**Authors:** Jian-biao Meng, Yan-na Jiao, Geng Zhang, Xiu-juan Xu, Chun-lian Ji, Ma-hong Hu, Zhi-zhen Lai, Ming Zhang

**Affiliations:** ^1^Intensive Care Unit, Tongde Hospital of Zhejiang Province, 234 Gucui Road, Hangzhou 310012, China; ^2^Intensive Care Unit, The First Affiliated Hospital, College of Medicine, Zhejiang University, 79 Qingchun Road, Hangzhou 310003, China; ^3^Intensive Care Unit, Hangzhou Cancer Hospital, 34 Yan Guan Lane, Hangzhou 310002, China

## Abstract

**Objective:**

To investigate the effects of electroacupuncture (EA) at “Zusanli” (ST36) and “Shangjuxu”(ST37) on reducing inflammatory reaction and improving intestinal dysfunction in patients with sepsis-induced intestinal dysfunction with* syndrome of obstruction of the bowels Qi*.

**Methods:**

A total of 71 patients with sepsis-induced intestinal dysfunction with* syndrome of obstruction of the bowels Qi* were randomly assigned to control group (n=36) and treatment group (n=35). Patients in control group were given conventional therapies including fluid resuscitation, anti-infection, vasoactive agents, mechanical ventilation, supply of enteral nutrition, and glutamine as soon as possible. In addition to conventional therapies, patients in treatment group underwent 20 minutes of EA at ST36-ST37 twice a day for five days. At baseline, day 1, day 3, and day 7 after treatment, the plasma levels of procalcitonin (PCT), tumor necrosis factor-*α* (TNF-*α*), intestinal fatty acid-binding proteins (I-FABP), D-lactate, citrulline, and TCM quantitative score of intestinal dysfunction were measured and recorded, respectively. And days on mechanical ventilation (MV), length of stay in intensive care unit (ICU), and 28d mortality were recorded.

**Results:**

During treatment, the plasma levels of PCT, TNF-*α*, I-FABP, D-lactate, and TCM quantitative score of intestinal dysfunction were declining in both groups, while the treatment group showed a significant decline (*P<0.05*). Plasma levels of citrulline were increasing in both groups, while the treatment group showed a significant increase (*P<0.05*). However, there were no significant differences in the days on MV, length of stay in ICU, and 28d mortality between two groups (*P>0.05*).

**Conclusions:**

EA at ST36-ST37 can reduce inflammatory reaction and has protective effects on intestinal function in patients with sepsis-induced intestinal dysfunction with* syndrome of obstruction of the bowels Qi*.

**Trial Registration:**

This trial was registered at http://www.chictr.org.cn/(ChiCTR-IOR-17010910).

## 1. Introduction

Sepsis is life-threatening organ dysfunction caused by a dysregulated host response to infection [1]. Despite advances in medical therapy and widespread adoption of international sepsis guidelines, sepsis is still a major global public health challenge and the mortality rate of patients with sepsis remains high [2, 3]. Sepsis is a complex entity and therapy for sepsis remains nonspecific outside of targeted antimicrobial therapy, resulting in trying to understand its underlying pathophysiology.

The gut has long been hypothesized to be “the motor” of critical illness and specific sepsis, driving systemic inflammation through a number of disparate feedback and feedforward mechanisms [4]. In order to maintain the blood supply of the vital organs during hemorrhagic shock, the intestinal blood flow sharply reduced, and dysfunction of the intestinal mucosal barrier occurs. The integrity of the intestinal barrier can be compromised in critically ill patients and specifically in septic patients [5, 6], manifesting intestinal ischemic injury, intestinal hyperpermeability, and intestinal barrier dysfunction. Intestinal barrier dysfunction is a highly severe condition, with a high mortality rate in patients with sepsis. For the lack of an available diagnostic biomarker, researchers have long sought to identify a biomarker or a combination of markers to ensure a specific, sensitive, and early diagnosis of intestinal dysfunction. Moreover, as shown in lots of diseases, the combination of several biomarkers rather than the use of a single marker is probably a better paradigm to investigate. Shi et al. showed that serum D-lactate levels were increased in acute intestinal ischemic injury patients, and the sensitivity of serum D-lactate ranged between 67% and 90%[7], whereas the specificity reached 87%. Many clinical studies showed a correction between the duration of ischemia and the increase of serum intestinal fatty acid-binding proteins (I-FABP) and a pooled sensitivity of 80% for serum I-FABP and a pooled specificity of 85% in the diagnosis of acute intestinal injury [8, 9]. In a clinical observation, Piton et al. evidenced that plasmatic citrulline concentration was shown to decrease in the first hours of shock in critically ill patients and was related to mortality within 28 days [10]. Therefore, I-FABP, D-lactate, and citrulline are promising candidate biomarkers.

Acupuncture, one of the therapeutic maneuvers in traditional Chinese medicine (TCM), has been applied in clinics for thousands of years, and it has been evidenced to have a bidirectional neuron-endocrine-immune system regulating effect and antagonize systemic inflammatory response without side-effects. According to TCM theory, the ST36 (*Zusanli*) and ST37 (*Shangjuxu*) acupuncture points are located at 3 and 6 cm, respectively, below the knee joint on the anterior aspect of the leg. In animal studies, Du M et al. found that electroacupuncture (EA) at ST36 relieved intestinal barrier injury and system inflammation in a rat ischemia model through activating the cholinergic anti-inflammatory pathway [11]. EA at ST36 may reduce the severity of acute pancreatitis by inducing anti-inflammatory effects and reducing the time to refeeding in patients with acute pancreatitis and EA at ST36 may accelerate the recovery of gastrointestinal motility after colorectal surgery [12, 13]. Wu J et al. indicated that electroacupuncture at ST36-ST37 improved the immunological function [14], decreased intestinal permeability[15], and recovered intestinal function in patients with sepsis[16]. EA also shortened period of recovery of bowel sound, improved the intestinal function, and reduced complications in postoperative patients[17].

During the clinical treatment of sepsis, oral Chinese medicine, acupuncture, and other traditional methods are applied to treat intestinal dysfunction of sepsis, and some effects have been obtained. However, the effects of EA at ST36-ST37 on sepsis-induced intestinal dysfunction with* syndrome of obstruction of the bowels Qi* remain unknown. Therefore, the aim of this study was to determine whether sepsis-induced intestinal dysfunction with* syndrome of obstruction of the bowels Qi* is improved with EA at ST36-ST37.

## 2. Materials and Methods

### 2.1. Ethics Statement

The study was conducted in accordance with the guidelines of the Declaration of Helsinki [18] and was approved by the Ethics Committee of Tongde Hospital of Zhejiang Province (approval no. [2015]051-018).

### 2.2. Settings and Patients

A target sample of 84 patients, aged 18-80 years, with sepsis-induced intestinal dysfunction with* syndrome of obstruction of the bowels Qi*, were recruited at Tongde Hospital of Zhejiang Province between March 2017 and October 2017. All the participants received treatment in the intensive care unit (ICU) of this hospital.

It was estimated that a sample size of 35 patients per group would be required for this preliminary study. To our knowledge, no similar study has been reported in the literature; thus, due to lack of baseline information about the potential discrepancy between* de qi* induced by needle manipulation and actual sensation of* de qi*, a more sophisticated power calculation was not possible. Group sizes were inflated to n=42 (total n=84 subjects), assuming a 20% dropout rate. Patients and study investigators were blind to allocation.

Sepsis was diagnosed according to the criteria outlined in the Surviving Sepsis Campaign: International Guidelines for Management of Sepsis and Septic Shock: 2016 published in the* Critical Care Medicine *[19], and intestinal dysfunction was diagnosed according to the criteria outlined in the gastrointestinal function in intensive care patients: terminology, definitions, and management [20], while the* syndrome of obstruction of the bowels Qi *pattern was diagnosed according to an expert consensus of diagnosis and treatment of integrated traditional Chinese and Western medicine on sepsis [21]. The* syndrome of obstruction of the bowels Qi* shows abdominal distension, abdominal distension as stiff as a drum, abdominal pain refusing to pressure, exhausting gas from anus frequent, coma and delirium, dry and yellow or burned black fur of tongue, and sunken and solid pulse [21].

All patients included in this study or their relatives consented to participation. All patients had at least a type of infection and were diagnosed to be sepsis. Patients had suffered from intestinal dysfunction and* syndrome of obstruction of the bowels Qi.* Patients with malignant tumor, pregnancy, fainting during acupuncture, infected sites of ST36, ST37, and inflammatory bowel disease were excluded from this study.

Every potential participant or relative was evaluated and informed about the procedures as well as the risks involved with participation in this study at the initial interview, and a full past medical history was taken. Candidates who went through the preliminary evaluation and signed consent underwent further examination and those who satisfied all the inclusion criteria were enrolled in the ICU. Baseline demographic data, including current age, sex, acute physiology, and chronic health evaluation (APACHE)-II, the delay between admission and inclusion, TCM quantitative score of intestinal dysfunction, and type of infection were collected.

### 2.3. Treatment Protocol

After completing the baseline evaluation, patients were randomly assigned to either the control group or the treatment group in a 1:1 ratio using a table of random numbers. In the control group, patients were given mechanical ventilation using a volume controlled mode with a tidal volume of 6 mL/kg of predicted body weight to attain acceptable blood gases and were provided with midazolam and fentanil for sedation and analgesia respectively, if necessary. And extubation was undertaken when indicated clinically. Extubation was performed when there was no evidence of being cardiovascularly unstable and having arterial oxygen tension (Pa0_2_) >80 mmHg on an inspired oxygen concentration (FiO_2_) <40% and a positive end-expiratory pressure (PEEP) <5 cmH_2_O. According to the protocol of Rivers et al. [22], patients with sepsis-induced tissue hypoperfusion were provided with adequate initial resuscitation. Daily fluid balance was recorded. Norepinephrine (3 to 40*μ*g/min) was given to maintain mean arterial pressure (MAP) at levels > 65 mmHg. The need for red blood cell (RBC) transfusion was determined based on the patient's hematocrit (HCT) concentration. Regular regimens were used in enteral nutrition; glutamine (0.2-0.4mg/kg/day) was provided intravenously in patients on parenteral nutrition. If patients could not self-defecate in 24 hours after enrolment, they were given nasogastric feeding of Dachenqi Decoction (50ml decoction made from 12g* Dahuang*, 24g* Houpu*, 12g* Zhishi*, and 6g* Mangxiao*) for twice a day until defecation. The periods from administration of Dachenqi Decoction to defecation were recorded. The TCM quantitative score of intestinal dysfunction (Table 1) were recorded at baseline and at the first, the third, and the seventh days in control group and treatment group.

In addition to therapies mentioned above, patients, in group treatment, were also provided with EA at ST36-ST37.

### 2.4. Electroacupuncture

Each patient in the treatment group received EA twice a day for five days. After conventional disinfection with iodine and alcohol, 0.30×40mm needles (Hwato, Suzhou, China) were inserted bilaterally 20-25mm beneath the skin at ST36 and ST37 with manual lift-thrust to elicit* qi* (a characteristic needing sensation perceived by the subject while the acupuncturist felt a needle grasp). Then the needles were connected to an EA stimulator (KWD-808I, Changzhou, China). Stimulation was performed using a continuous wave, a frequency of 4Hz, and the intensity was adjusted to induce visible muscle twitching for the duration of the 20-min EA period.

### 2.5. Measurement

Assessment was undertaken at baseline and at the first, the third, and the seventh days, with measurement of biomarkers plasma levels of intestinal dysfunction (I-FABP, D-lactate, and citrulline) and plasma levels of inflammatory factors (procalcitonin, PCT and tumor necrosis factor-*α*, and TNF-*α*).

Blood samples were drawn at baseline and at 1, 3, and 7 days. Plasma samples were immediately placed at room temperature for 10 minutes and then centrifuged at 3,500 rpm for 15 minutes (80-2 centrifuge; Changzhou Guoyu Instrument Manufacturing Co., Ltd. China.). Samples were then decanted and placed in 5-ml collection tubes and stored in a monitored −80°C specimen freezer until analysis was performed. Citrulline concentrations were determined by high performance liquid chromatography (HPLC) using the Hitachi L-8800 Amino Acid Analyzer (Tokyo, Japan). Plasma I-FABP and D-lactate levels were measured using enzyme-linked immunosorbent assay (ELISA) kits (R&D Systems, Minneapolis, USA) according to the manufacturer's instructions.

After samples were collected, they were centrifuged at 2,000 rpm for 15 minutes and stored in a freezer at −20°C until they were ready for processing and analysis. The ELISA kits (ExCell Biology, Shanghai, China) were used to determine the levels of TNF-*α* in the samples and the data were analyzed. All the samples were discarded after the analysis.

Blood samples were drawn and sent to the laboratory (Tongde Hospital of Zhejiang Province, Hangzhou, China) for detection the levels of PCT.

### 2.6. Statistical Analyses

The statistical analyses were performed by a researcher who is blinded to the allocation. Following the per protocol (PP) principle, all the data were analyzed using SPSS software (version 19.0, SPSS Inc., Chicago, IL, USA) and the results were presented as mean ± standard deviation (SD) or number (%).

Distributions of the discrete variables were compared between the two treatment groups with either the Chi-square test or Fisher exact tests. Two-sample* t*-test was used to compare between the two groups and SNK-*q* test to compare continuous variables before and after treatment. all tests were 2-tailed and* P *< 0.05 was considered to be statistically significant.

## 3. Results

### 3.1. Patient Enrolment

During the period of recruitment from March 2017 to October 2017, 134 patients received a preliminary diagnosis of sepsis (Figure 1). A total of 30 patients were excluded because they did not meet the formal diagnostic criteria for sepsis-induced intestinal dysfunction, and 20 relatives of patients did not sign consent. Finally, 84 patients with sepsis-induced intestinal dysfunction with* syndrome of obstruction of the bowels Qi *were enrolled in the study. 13 patients were found to have been erroneously included as giving up treatment (six in the control group and seven in the treatment group) during period of the trial and were therefore excluded from the primary statistical analysis. As a result, data from 71 participants were analysed.

### 3.2. Baseline Data

The demographic data were not significantly different between the control group and treatment group(Table 2): 59.8±13.3 versus 61.7±14.9 years old (age;* P *= 0.560); 19 versus 16 males (*P *= 0.552). The assessment score and TCM quantitative score of intestinal dysfunction at admission were not significantly different between the control group and the treatment group: 18.1±3.9 versus18.9±4.2 (APACHE II score;* P *= 0.391); 10.5±3.0 versus 9.8±2.7 (TCM quantitative score of intestinal dysfunction;* P *= 0.901. The delay between admission and inclusion in two groups was 12.8±5.1 versus 11.9±4.8 (*P *= 0.896). The sites of infection which contributed to intestinal dysfunction in all patients included lung, abdomen, bloodstream, and urinary tract and none of them showed significant difference. The use of Dachenqi Decoction was similar between the control group and treatment group: 29(80.6%) versus 26(74.3%) (*P *= 0.527). In the treatment group, however, the periods from administration of Dachenqi Decoction to defecation were less than the control group: 20.2±2.4 versus 15.8±2.6 hours (*P *= 0.001) (Table 2).

### 3.3. Changes in Biomarkers Plasma Levels and TCM Quantitative Score of Intestinal Dysfunction

There were no significant differences in plasma levels of I-FABP, D-lactate, citrulline, and TCM quantitative score of intestinal dysfunction at baseline between two groups (*P *= 0.394, 0.692, 0.222, 0.901, respectively). During the course of treatment, plasma levels of citrulline increased gradually while I-FABP and D-lactate decreased in two groups, but citrulline increased more significantly at day 1, day 3, and day 7 in the treatment group versus the control group (*P =0.001,* <0.001, <0.001, respectively); moreover, I-FABP and D-lactate decreased more significantly at day 1, day 3, and day 7 in the treatment group versus the control group (all* P *<0.001). After treatment, although TCM quantitative score of intestinal dysfunction decreased in two groups, they decreased more significantly at day 3 and day 7 in the treatment group versus the control group (*P *= 0.042, 0.016 respectively) (Table 3).

### 3.4. Changes in Plasma Levels of Inflammatory Factors

There were no significant differences in plasma levels of PCT and TNF-*α* at baseline between two groups (*P *= 0.563, 0.921, respectively). After treatment, although the plasma levels of PCT and TNF-*α* decreased in two groups, PCT and TNF-*α* decreased more significantly at day 1, day 3, and day 7 in the treatment group versus the control group (*P *= 0.017, 0.014, 0.002 respectively, PCT;* P* <0.001, <0.001, =0.001, respectively, TNF-*α*.) (Table 4).

### 3.5. Prognosis

Compared to patients in the control group, days on MV and length of stay in ICU were not shortened significantly in the treatment group(8.3±2.1 versus 7.7±2.0 days,* P* =0.260, days on MV and 13.9±2.7 versus 13.6±2.8,* P* =0.601, length of stay in ICU). And the overall mortality at day 28 did not show significant difference between two groups (41.7% versus 37.1%, resp.,* P* = 0.697).

### 3.6. Safety of Acupuncture

No adverse effects of acupuncture were documented during the study.

## 4. Discussion

The present study was designed to investigate the protective effect of EA at ST36-ST37 in patients with sepsis-induced intestinal dysfunction with* syndrome of obstruction of the bowels Qi*. Comparing the treatment group (n=35), in which patients were expected to experience EA at ST36-ST37 by design, with the control group (n=36), in which no EA at ST36-ST37 was expected, there were no significant differences in overall mortality at day 28 and both groups showed similar days on MV and length of stay in ICU, suggesting the prognosis was not improved by EA at ST36-ST37. Superficial examination of our results may lead to a hasty conclusion that EA at ST36-ST37 is irrelevant for the protection in patients with sepsis-induced intestinal dysfunction with* syndrome of obstruction of the bowels Qi*. However, as is shown in the study, EA at ST36-ST37 not only improved intestinal function but also decreased inflammatory reaction in patients with sepsis-induced intestinal dysfunction with* syndrome of obstruction of the bowels Qi*.

Sepsis is life-threatening organ dysfunction caused by a dysregulated host response to infection [1]. The occurrence of it is due to a variety of injuries caused by the release of inflammatory mediators or ischemia reperfusion injury, which can injure intestinal mucosal barrier function, result in the translocation of bacteria, endotoxin, and various kinds of metabolites, and, as a result of the enterogenous bacteremia, eventually lead to or exacerbate sepsis and multiple organ dysfunction syndrome (MODS). Therefore, intestinal dysfunction is not only a result but a trigger in the pathogenesis of sepsis and MODS. In TCM, according to the intestinal typing of sepsis, sepsis and MODS are divided into four types including* excessive heat syndrome, syndrome of blood stasis, syndrome of exhaustion, and syndrome of obstruction of the bowels Qi. The syndrome of obstruction of the bowels Qi *manifests intestinal dysmotility and intestinal barrier dysfunction in clinical, which are in accordance with manifestation of intestinal dysfunction[23]. Hence, sepsis-induced intestinal dysfunction with* syndrome of obstruction of the bowels Qi was selected in this study.*

During sepsis and septic shock, the effects of sepsis and ischemia can coexist when splanchnic hypoperfusion occurs [24], and it has been postulated that intestinal may be contribute to the subsequent development of sepsis [25]. PCT and TNF-*α* are the important biomarkers of infection and inflammation, and elevated levels of PCT and TNF-*α* are usually related to the severity and poor prognosis of sepsis [26–29]. In this study, the results indicated that EA at ST36-ST37 exert its anti-inflammatory effects mainly by decreasing PCT and TNF-*α* in plasma. However, though the markers show acceptable sensitivities, in certain degree, none of them are specific enough to be used as a diagnostic marker of sepsis and sepsis-induced intestinal dysfunction.

As the pathophysiology of sepsis-induced intestinal dysfunction involves intestinal insufficiency, ischemic injuries, mucosal tissue injury, and loss of enterocyte mass [30], compared to PCT and TNF-*α*, I-FABP, D-lactate, and citrulline might be more promising candidate biomarkers related to the pathophysiology of ischemia, intestinal insufficiency, and gut barrier failure [31–34]. And they were selected to assess sepsis-induced intestinal dysfunction with* syndrome of obstruction of the bowels Qi. *As is shown in the study, EA at ST36-ST37 decreases plasma levels of I-FABP and D-lactate and increases citrulline.

In this study, patients with sepsis suffered from* syndrome of obstruction of the bowels Qi* which were manifested as abdominal distension, emesis, none of defecation and evacuation, and hypoactive bowel sounds. And TCM quantitative score of intestinal dysfunction in sepsis-induced intestinal dysfunction with* syndrome of obstruction of the bowels Qi* was increased in our study and EA at ST36-ST37 significantly reduced the TCM quantitative score of intestinal dysfunction. Although there were no differences in the number of patients given Dachenqi Decoction between two groups(*P *= 0.527), the periods from administration of Dachenqi Decoction to defecation in the treatment group were significantly shorter than in the control group. Hence, EA at ST36-ST37 contributes to reduction in the period of defecation and even the usage of Dachenqi Decoction. It is accepted that the gut is not only the key organ but the amplifier of mediators of inflammation. Therefore, it is the most important to adopt purgative therapy to keep the gut to be unobstructed in patients with sepsis-induced intestinal dysfunction with* syndrome of obstruction of the bowels Qi. *And blockade or decreasing the injury in intestines and production of proinflammatory mediators should be considered as the main methods to protect intestines and reduce the inflammatory response in sepsis.

ST36 and ST37 are the points of the Stomach Meridian of Foot-Yangming, ST36 is the confluent point of the Stomach Meridian of Foot-Yangming, and ST37 is the lower confluent point of the Large Intestine Meridian of Hand-Yangming. And their principle therapeutic indications are for diseases of digestive system, by exerting the effects of dredging the excretory organs and immunoregulation. Wu et al. indicated that EA at points of the Stomach Meridian of Foot-Yangming could cut down the plasma levels of TNF-*α* and IL-6 and inhibit the progression of inflammatory reaction in patients with sepsis [14]. Wang et al. showed that EA at ST36- ST 37 could shorten recovery time of bowel sound, accelerate defection, and facilitate recovery of gastrointestinal function in patients suffered abdominal surgical procedures [17]. In addition, EA at ST36- ST 37 could relieve constipation and expel toxin through dredging meridian, regulating pure and turbid of the spleen and stomach, up and down of Qi Movement, coordinating yin yang, strengthening body resistance, and fostering foundation of life [35]. It was also found that EA at ST36 could improve gastrointestinal barrier of mucous membrane through ameliorating neural regulation, regulating secretion of gastrointestinal hormone, enhancing blood supply of gastrointestinal mucous membrane, and cleaning inflammatory mediator [36]. However, the mechanism of anti-inflammatory and protection of gut in septic patients is still unclear. In previous study conducted by Borvikova et al., “cholinergic anti-inflammatory pathway” was named, and it could antagonize proinflammatory factors directly and alleviate the lethal effect of endotoxin. In cholinergic anti-inflammatory pathway, it was considered that pathway of cholinergic nerve and its neuro-transmitter-acetylcholine (ACh) regulated systemic inflammation [37]. EA at ST36 had a significant effect on central nuclei of the vagus nerve including dorsal nuclei of vagus nerve, solitary tract, nucleus of solitary tract, and ambiguous nucleus [38]. The afferent somatic messages from ST36-ST37 by EA at them could be transmitted to nucleus of solitary tract, which affect the motor activity of the stomach and gut and electrical release by efferent vagus nerve [39]. In our study, EA at ST36-ST37 showed anti-inflammatory and gut protection, which may be attributed to release of Ach by the vagus nerve as a result of transmission of message to vagus nuclei consequent on EA of ST36-ST37 acupoints and the bilateral division of vagus nerve. The mechanism of EA is very complicated and unclear; however, activation of cholinergic anti-inflammatory pathway may be considered to be one of the main mechanisms of EA at ST36-ST37, exerting the effect of anti-inflammation and improving* syndrome of obstruction of the bowels Qi* and protective effect on intestinal function in patients with sepsis-induced intestinal dysfunction with* syndrome of obstruction of the bowels Qi.*

In our study, however, there were no significant differences in days on mechanical ventilation, length of stay in ICU, and 28-day mortality between two groups. The reasons maybe as follows. First, lower immunocompetence, more underlying diseases, and higher complications resulted in higher mortality in patients with sepsis-induced intestinal dysfunction with* syndrome of obstruction of the bowels Qi*, and the improvement in intestinal function is still inadequate to affect the progress of pathogenetic progression and inverse the prognosis in these patients. Second, this study is a small sample size and single-center investigation and may not represent results for the general population completely. Further investigations are, therefore, required to refine our technique and expand sample size.

## 5. Conclusions

In conclusion, in addition to their anti-inflammatory effects mainly by decreasing PCT and TNF-*α* in plasma, EA at ST36-ST37 also showed to able to decrease I-FABP and D-lactate and enhance citrulline in plasma, and improve* syndrome of obstruction of the bowels Qi,* indicating that they were able to exert a protective effect on intestinal function in patients with sepsis-induced intestinal dysfunction with* syndrome of obstruction of the bowels Qi.*

## Figures and Tables

**Figure 1:** Diagram of the study.

**Table 1:** TCM quantitative score of intestinal dysfunction.

Item	Score			
	0	1	2	3
Abdominal distension	None	Mild abdominal distension	Moderate abdominal distension with tolerance	Severe abdominal distension without tolerance
Diarrhea(times/day)	None	3-4	5-10	>10
Bowel sounds	Normal	Hyperactive or weakened	Significantly weakened or decrease	All disappeared
Weight loss	None	<10%	>10% and <20%	>20%
Defecation	Self -defecation in 24 hours	No self-defecation in 24 hours	No self-defecation in 24 hours after oral/nasogastric feeding of cathartic	No self-defecation in 48 hours after oral/nasogastric feeding of cathartic or 24hours after enema
Fever (body temperature)	None	37.1-37.9°C	38.0-38.5°C	*⩾*38.6°C
Cyanosis	None	Mild cyanosis	Obviously cyanosis	cyanotic lips and nails

**Table 2:** Baseline characteristics of participants.

characteristics	Group control (n=36)	Group treatment (n=35)	*P*-Value
Age(years)	59.8±13.3	61.7±14.9	0.560
Male (n,%)	19(52.8%)	16(45.7%)	0.552
APACHEII	18.1±3.9	18.9±4.2	0.391
TCM quantitative score of intestinal dysfunction	10.5±3.0	9.8±2.7	0.901
Delay between admission and inclusion(hours)	12.8±5.1	11.9±4.8	0.896
Type of infection (n, %)			
Pneumonia	16(44.4%)	18(51.4%)	0.556
Peritonitis	7(19.4%)	7(20.0%)	0.953
CRBSI	6(16.8%)	4(11.4%)	0.526
Urinary tract infection	7(19.4%)	6(17.2%)	0.802
Dachenqi Decoction (as needed)			
Patients administrated ≥ 1 dose (n, %)	29(80.6%)	26(74.3%)	0.527
The periods from administration of Dachenqi	20.2±3.4	15.8±2.6	0.001
Decoction to defecation (hours)			
Days on MV	8.3±2.1	7.7±2.0	0.260
Length of stay in ICU(days)	13.9±2.7	13.6±2.8	0.601
28-day mortality% (n)	41.7%(15)	37.1%(13)	0.697

APACHE II: acute physiology and chronic health evaluation; CRBSI: catheter related bloodstream infection; MV: mechanical ventilation; ICU: intensive care unit.

**Table 3:** Serum markers and TCM quantitative score of intestinal dysfunction at different points in each group ($\overset{-}{\chi }$±*s*).

		Group control (n=36)	Group treatment (n=35)	*P*-Value
IFABP (ng/ml)	Baseline	71.48±14.69	68.62±13.39	0.394
	Day 1	56.29±14.64^#^	44.42±10.26^#^	0.001
	Day 3	40.55±10.87^#*∗*^	21.38±6.98^#*∗*^	0.001
	Day 7	23.16±6.27^#*∗*△^	12.67±5.27^#*∗*△^	0.001
D-lactate (mmol/L)	Baseline	6.16±1.30	6.03±1.56	0.692
	Day 1	4.55±1.55^#^	3.23±1.10^#^	0.001
	Day 3	3.69±1.65^#^	1.80±1.03^#*∗*^	0.001
	Day 7	2.24±0.66^#*∗*△^	1.33±0.43^#*∗*△^	0.001
Citrulline (*μ*mol/L)	Baseline	9.41±3.98	8.15±4.63	0.222
	Day 1	13.90±3.80^#^	17.07±4.02^#^	0.001
	Day 3	14.85±3.80^#^	20.50±4.52^#*∗*^	0.001
	Day 7	18.53±4.67^#*∗*△^	25.28±4.97^#*∗*△^	0.001
TCM quantitative score of intestinal dysfunction	Baseline	10.5±3.0	9.8±2.7	0.901
	Day 1	9.9±2.8	8.7±2.6	0.066
	Day 3	9.1±2.9^#^	7.6±3.2^#^	0.042
	Day 7	8.2±1.9^#*∗*^	6.9±2.5^#*∗*^	0.016

IFABP: intestinal fatty acid binding protein; TCM: Traditional Chinese Medicine.

# *P<0.05* relative to baseline; *∗*  *P<0.05 *relative to day 1; △  *P<0.05 *relative to day 3.

**Table 4:** Levels of serum inflammatory factors at different points in each group ($\overset{-}{\chi }$±*s*).

		Group control (n=36)	Group treatment (n=35)	*P*-Value
PCT (ng/ml)	Baseline	7.45±3.41	6.98±3.45	0.563
	Day 1	5.34±2.99^#^	3.75±2.45^#^	0.017
	Day 3	3.39±2.68^#*∗*^	2.01±1.83^#*∗*^	0.014
	Day 7	2.90±1.83^#*∗*^	1.54±1.80^#*∗*^	0.002
TNF-*α*(pg/ml)	Baseline	93.64±27.67	94.33±29.87	0.921
	Day 1	85.22±25.59	58.81±20.63^#^	0.001
	Day 3	67.74±30.66^#^	33.64±18.53^#*∗*^	0.001
	Day 7	34.13±21.08^#*∗*△^	19.68±11.70^#*∗*△^	0.001

PCT: procalcitonin; TNF: tumor necrosis factor.

# *P<0.05* relative to baseline; *∗*  *P<0.05 *relative to day 1; and △  *P<0.05 *relative to day 3.

## Data Availability

The data used to support the findings of this study are available from the corresponding author upon request.
